# Optimization of a Deep Learning Algorithm for Security Protection of Big Data from Video Images

**DOI:** 10.1155/2022/3394475

**Published:** 2022-03-08

**Authors:** Qiang Geng, Huifeng Yan, Xingru Lu

**Affiliations:** ^1^School of Big Data & Software Engineering, Chongqing College of Mobile Communication, Chongqing 401520, China; ^2^Chongqing Key Laboratory of Public Big Data Security Technology, Chongqing 401420, China; ^3^School of Software Engineering, Chongqing University of Posts and Telecommunications, Chongqing 400065, China

## Abstract

With the rapid development of communication technology, digital technology has been widely used in all walks of life. Nevertheless, with the wide dissemination of digital information, there are many security problems. Aiming at preventing privacy disclosure and ensuring the safe storage and sharing of image and video data in the cloud platform, the present work proposes an encryption algorithm against neural cryptography based on deep learning. Primarily, the image saliency detection algorithm is used to identify the significant target of the video image. According to the significant target, the important region and nonimportant region are divided adaptively, and the encrypted two regions are reorganized to obtain the final encrypted image. Then, after demonstrating how attackers conduct attacks to the network under the ciphertext attack mode, an improved encryption algorithm based on selective ciphertext attack is proposed to improve the existing encryption algorithm of the neural network. Besides, a secure encryption algorithm is obtained through detailed analysis and comparison of the security ability of the algorithm. The experimental results show that Bob's decryption error rate will decrease over time. The average classification error rate of Eve increases over time, but when Bob and Alice learn a secure encryption network structure, Eve's classification accuracy is not superior to random prediction. Chosen ciphertext attack-advantageous neural cryptography (CCA-ANC) has an encryption time of 14s and an average speed of 69mb/s, which has obvious advantages over other encryption algorithms. The self-learning secure encryption algorithm proposed here significantly improves the security of the password and ensures data security in the video image.

## 1. Introduction

The development of the fifth-generation mobile communication system promotes the advent of the era of Internet of Things (IoT). People's production and life are inseparable from IoT technology. A variety of information sensing devices are combined with a large-scale network to form a real-time interconnection between real things and computers in the case of uncertain time and place [1, 2]. In the process of information transmission, there are many videos and images generated. These video images contain a large amount of people's private information. If information of these video images is not encrypted before information transmission, it is very likely to cause severe damage to personal privacy and even affect the overall interests of a group of network users [3, 4]. Therefore, the protection of video image data security has become a key concern for recent research studies. Protecting the security of big data from video images can effectively avoid the problem of user privacy disclosure, to ensure the safe storage and transmission of video images in the cloud platform [5].

The method of encrypting the video image is to make the semantic information in the video image chaotic so that it cannot be easily obtained by cyber hackers. Concurrently, even if the attackers successfully obtain the ciphertext images, they cannot get effective information from them, and the receiver of the video image will obtain the key in advance to recover the original video image. In recent years, scholars have proposed a variety of video image encryption algorithms such as compressed sensing, DNA coding, optical conversion, and chaotic system. Different data encryption algorithms also have different characteristics, and the amount of calculation and encryption effect is also different. Li et al. (2020) [6] proposed a real-time video secure communication system based on a new grid multiwing chaotic system to study the application of the chaotic system in video image encryption. Compared with the existing multiscroll and multiwing chaotic system, it is found that the system has a simple structure and is easy to be realized in the digital system. The feasibility is verified by specific experiments. Additionally, through a series of widely used safety analyses, it is proved that the system has good safety performance. Panwar et al. (2021) [7] proposed a fast and secure image encryption technology. The encryption scheme is designed to securely transmit video surveillance data on an insecure network. Image encryption technology adopts a one-dimensional sinusoidal system, which has better chaotic characteristics than seed mapping and is faster than the high-dimensional chaotic system. Besides, the design of the encryption scheme is based on two rounds of replacement, adopts simple pixel exchange operation and diffusion operation, and provides the security required for plaintext, differential, and various other attacks [8, 9].

However, by consulting relevant literature, it is found that the current encryption methods for video image data are mainly designed for important areas. However, they do not carry out encryption protection and further information compression for nonimportant areas. Here, the study is carried out on an encryption algorithm ANC (advantageous neural cryptography) based on an antineural network. Trying to alleviate the shortcomings of the algorithm, the present work develops an improved encryption algorithm CCA-ANC based on theories about the chosen ciphertext attack (CCA). The model constructed here has the following advantages: (1) it can make corresponding defense schemes through the attacker's attack behavior to ensure the security of the key; (2) because of the competition among the data sender, the legitimate data receiver, and the attacker, the resulting encryption algorithm can resist robust decoding and calculation; (3) it constructs a security detection network structure to analyze the security degree of the transmitted data; (4) it can ensure the integrity of the communication data and the accuracy of the received recovery data as far as possible under the premise that it can resist decipherers.

## 2. Relevant Research and Analysis

### 2.1. Development History and Current Situation of Video Image Encryption

The purpose of image encryption is to disrupt the semantic information of the image so that the attacker cannot obtain valid information after intercepting the ciphertext image. The legitimate receiver can still restore the original image through the agreed key and public encryption and decryption algorithm. In recent years, researchers have proposed many encryption algorithms, including chaotic systems, optical transformations, aeoxyribonucleic acid (DNA) coding, compressed sensing, and other encryption technologies. Different encryption algorithms have different characteristics, encryption effects, and computation volumes. According to the characteristics of the encryption algorithm, it can be divided into spatial encryption and frequency domain encryption. The spatial encryption's main idea is to conduct scrambling and diffusing on the image: scrambling refers to changing the pixel value, and diffusion is to scramble the pixel's position.

A sine function is innovatively introduced in exploring image encryption to propose a new one-dimensional chaotic system image encryption scheme. It makes the chaotic phenomenon of the chaotic system more prominent and enhances the image encryption effect. However, its encryption strength for critical data is insufficient and cannot ensure data security. A high-order chaotic system is introduced into the image encryption scheme to ensure the security of encrypted data. In addition, DNA coding processes data in parallel and contains a large amount of information. Because fixed encoding rules cannot be applied to the encryption system as an independent technology, a scheme combining a high-dimensional chaotic system with DNA encoding is proposed to enhance the encryption strength and the security of the encrypted image. However, the encryption methods mentioned above mainly focus on the security and encryption performance but ignore the compression of images. As an image processing method, compressed sensing can compress or encrypt images and save storage resources and protect images. The basic idea of compressed sensing is to compress the sparse signal with a perception matrix and then reconstruct the original signal by solving a convex optimization problem. However, due to the insufficient security of compressed sensing technology, it is generally not used in heavy encryption. Instead, some traditional encryption methods are applied to compressed sensing technology.

The early video encryption scheme regarded the encoded video as a bit stream and encrypted it with traditional methods, such as advanced encryption standard (AES). This method of encrypting only the bit stream is called the naive encryption algorithm. It is not applicable to any syntax elements and unique structures but only treats high efficiency video streams as text data. At present, there is no algorithm to crack triple AES, so AES can provide high security for videos.

In the process of video encoding and decoding, the syntax elements after entropy encoding play a vital role in the reconstruction of video frames, which will affect the quality of the final encoded video. The choice of the encryption algorithm is to encrypt some essential syntax elements after video entropy coding so that the video is seriously distorted to achieve the effect of video encryption. The video with encrypted video syntax elements will be severely distorted after decoding so that the reconstructed video cannot obtain any useful information, and the user who holds the key can obtain the original video.

### 2.2. Pivotal Technology of Neural Networks in Cryptography

Designing a cryptographic system based on neural networks is complex system engineering. Cryptographic designers need to understand key technologies such as the topology of neural networks and need knowledge of weighted adaptive iteration and encryption and decryption systems. The bit error rate in the cryptosystem based on a neural network is as low as possible to ensure security. Applying neural networks in cryptography requires many necessary artificial neural network technologies.

1. Tree parity machine (TPM) is used to exchange the synchronization state on the input and output of both parties as a key and exchange keys through a public channel to generate a public key system
2. Chaotic logic mapping neural network is used in cryptography. Both parties use the neural network as the input of the logic mapping to generate the output bits to be learned
3. General regression neural network (GRNN) is used to perform the encryption and decryption process based on three layers, in which the input data is 3 bits, and the output data is 8 bits
4. Backpropagation is trained to be the public key, and the Boolean number is trained as the private key
5. A time-varying time-delay chaotic hopfield neural network (CHNN) is used to generate a binary sequence and encrypt it as a random switching function of the chaotic map
6. The chaotic dynamic behavior generated by the neural network based on the chaotic generator is used as the public key
7. The pseudorandom number (PRN) generator based on neural networks is used as a key generator in a stream cipher
8. The chaotic neural network is used to generate chaotic sequence as the tripartite key of cryptography (the initial condition and control parameters are combined)
9. The weight matrix of layer recurrent neural network (LRNN) is used to generate pseudorandom numbers as keys
10. The initial weight of the trained neural network is used as a symmetric key

In addition, other techniques can be applied in cryptography, and different techniques have different effects.

### 2.3. Application of Neural Networks in Cryptography

As neural networks are used in increasingly tricky projects, they are trained to meet the goals of simple functions and solve complex problems, including generating realistic images and solving multiagent issues. While promoting these works, neural networks can learn to protect their communication security by coping with the strategies of specific opponents.

Cryptography involves many aspects; the most important of which is the design of algorithms and structures to ensure data security and data integrity. Cryptographic structures generally refer to assemblies or turing machines. Decipherers often use these terms to describe that the complexity of an algorithm (e.g., bounded in polynomial time) and the probability of success (e.g., bounded to a negligible probability) are limited. A security mechanism is considered secure if it can defend against all targets targeted by decipherers. For instance, if the decipherer cannot extract plaintext or critical information from encrypted data, this mechanism is safe. Modern cryptography provides this definition of security.

Decipherers also play an important role in designing and training neural networks. They frequently appear in adversarial examples and research on generative adversarial networks (GANs). In GANs, a decipherer is a particular class of the neural network that guesses whether the given data are constructed algorithmically or given from actual informative features. This method is different from the encryption method in cryptography theory. The actual design of GANs does not involve all the decoders in a category but uses training to resist some decoders. This paper utilizes these concepts as the design direction.

Different classes of neural networks are being used even more widely for problems related to cryptography. The current application of neural networks in cryptographic systems can be summarized into three parts.

#### 2.3.1. Synchronous Neural Networks

The mentioned artificial neural network used in the public channel to transmit the key comprises two multilayer neural networks, which can achieve synchronization using the mutual output bits as the training object. The experimental results show that the model will be faster, simpler, and more stable. The model has two neural networks in the public key encryption scheme based on neural networks. The system connects the neural network with the logical chaotic map. It also starts from different initial conditions through chaotic synchronization and alternately trains their output to synchronize to an equal time-related weight vector. Applying chaotic synchronization to neural cryptography can enhance the performance of cryptographic systems and improve security.

In the neural encryption key based on synchronous mutual learning of the tree parity check machine, the system has two identical dynamical systems aimed at different initial conditions and is synchronized by coupling to the common input value of the two systems. This model solves the security problem of numerical attacks. The general key generation method based on neural networks has two neural networks. They use the same characteristic input to generate an output bit and are trained according to it. If the outputs of both parties match, the weights can be modified, and the modified weights act as keys for the encryption and decryption process after synchronization. Simulation results indicate that the encryption algorithm based on neural networks is secure.

#### 2.3.2. Chaotic Neural Network

Chinese scholars have analyzed the encryption technology based on the time-varying delay-varying CHNN. The plaintext is encrypted by switching a chaotic neural network and the arrangement of binary data. The simulation results demonstrate that the chaotic encryption algorithm has excellent security performance in transmitting large multimedia files on public data communication networks. However, since the keystream used in each encryption process is the same, a chosen-plaintext attack can quickly obtain the keystream using two pairs of plaintext and ciphertext. The experimental analysis suggests that the chaotic cryptosystem designed here is insecure. Thus, a three-key chaotic neural network for image cryptography is proposed. Triple parameters are used to perform various operations on images to disrupt data in a seemingly random but actually specific sequence. Simulation analysis shows that this structure can generate secure passwords and can be applied to different color image sizes.

There are two main types of artificial neural networks used in cryptography. The first network is a neural network-based state sequence machine, and the other is a chaotic neural network. The first network uses a simple recurrent neural network based on a backpropagation training algorithm to generate a finite-state sequence machine whose startup state can be used as a key for encryption and decryption processes. The second network divides the message into multiple blocks, determines the initial value and control parameters, generates a chaotic sequence, and determines the parameters of the neural network based on the chaotic sequence as the key for the encryption and decryption process. Simulation analysis proves that the above network is safe and has high encryption efficiency.

#### 2.3.3. Multilayer Neural Network

The generalized regression neural network for the cryptography algorithm has a three-layer structure, and each layer has many primary neurons. The algorithm converts the input message into a 3 bit message set and generates 8 bit encrypted information after encryption. The experimental analysis shows that the encryption effect of the above algorithm is better than the traditional encryption method. Then, an asymmetric cryptographic mechanism is proposed based on a neural network. The creation process of the encryption and decryption scheme and the public key system depends on a multilayer neural network trained by the backpropagation learning algorithm. The encryption scheme and the private key creation process are based on Boolean algebra. Encryption systems are not based on number-theoretic functions and have lower time and memory complexity. The experimental results show that this model's security effect and encryption efficiency are equal to or better than the traditional methods.

In the electronic communication data security method based on neural networks, the neural network model converts ordinary information into a binary form and applies the neural network model to obtain different password information sequences. The simulation results demonstrate that the encryption structure based on the neural network has superior efficiency and security capability and can be used in real-time applications. Using the numerical solution of Chua's circuit, a neural network model is established for the chaotic cryptographic model based on the synchronization of a neural network and a chaotic generator. The simulation results prove that the model is efficient, safe, and reliable and can be applied to real-time applications. New modifications to the advanced encryption standard (AES) using nonlinear neural networks make the algorithm immune to specific attacks. The neural network model performs cryptographic processing through a symmetric key used as the initial weight of the neural network and is trained to obtain a fast and low-cost algorithm for its final weight. The simulation results show that the neural network-based AES cryptosystem proposed here is close to the results of the normal AES cryptosystem.

The neural network-based pseudorandom number generator model has high statistical security for key sequences. This neural pseudorandom number generator is a long series of patterns created by complete equations and initial values. The most prominent feature of these patterns is randomness. Simulation analysis suggests that the encryption system based on the neural network has high efficiency and is suitable for hardware applications.

## 3. Improved Generative Adversarial Network by CCA

Artificial intelligence (AI) research has achieved remarkable outcomes in recent years. At present, many artificial intelligence systems have made incredible breakthroughs in tasks such as image recognition, speech recognition, car driving, and intuitive games. Similarly, a crucial question in information security is whether AI will design or crack cryptographic algorithms better than human beings one day. Some papers in the literature try to use machine-learning techniques to design new cryptographic algorithms, and most of these works propose encryption schemes designed using the neural network as a tool to create nonlinearity. According to the literature, these schemes do not belong to AI because they are not based on the concept of security; in addition, with the demonstration of experienced cryptographic experts, these algorithms have proved to be seriously damaging to security.

In 2016, Abadi and Andersen of Google AI proposed a different encryption method, namely, ANC, in which there are three encryption and decryption agents: Alice, Bob, and Eve, who are in the encryption, decryption, and deciphering, compete with each other. Eve is a neural network trying to decipher Alice and Bob's communication data; Alice and Bob are also neural networks trying to learn how to protect their communication from Eve. Since Alice and Bob are in a state of self-taught security knowledge, their encryption method is different from other encryption methods. However, for the encryption algorithm they learned, there is a problem that they use a complex convolutional neural network but do not show what cryptographic system their system has learned, and they cannot judge whether it is a secure cryptographic structure. Security to another neural network does not mean absolute security. This paper proposes an improved ANC method using the concept of a CCA to overcome these limitations, resulting in the CCA-ANC. The main contribution of this paper is to demonstrate that AI can learn secure cryptographic algorithms without requiring human knowledge.

### 3.1. Nonequivalent Image Encryption Method

#### 3.1.1. Identification of Important/Nonimportant Areas

Here, the video image data is recognized based on the saliency detection model. In this detection model, the color, intensity, and direction of saliency mapping can be calculated by the difference between adjacent pixels and multiscale center. Then, the final saliency map is obtained by combining the above three feature maps [10–12].  Figure 1 demonstrates the specific algorithm steps.

**Step 1 .**

The intensity, color, and texture are adjusted according to the discrete cosine transform (DCT) coefficients of each 8∗8 block (*T*, *C*_*rg*_, *C*_*by*_) and other features to complete the construction of the feature map [13].

**Step 2 .**

The feature difference between each DCT block can be calculated as follows:

(1) $$\begin{array}{c} D_{m,n}^{r}=\zeta_{m}^{r}-\zeta_{m}^{r}. \end{array}$$

In the above equation, *r* represents the strength (*r*=1,2,3).

In DCT, equation (2) is used to determine the texture difference *D*_*m*,*n*_ between blocks *m*,  *n*:

(2) $$\begin{array}{c} D_{m,n}^{4}=max\left(P\left(U_{m},U_{n}\right),P\left(U_{m},U_{n}\right)\right). \end{array}$$

In the above equation, *U*_*m*_ denotes the text feature vector of the block *m*, and *U*_*n*_ indicates the texture feature vector of the block *n*. Equation (3) demonstrates the calculation method of *P*(*U*_*m*_, *U*_*n*_):

(3) $$\begin{array}{c} P\left(U_{m},U_{n}\right)=\underset{u_{m}\in U_{m}}{max}\underset{u_{n}\in U_{n}}{min}U_{m}-U_{n}. \end{array}$$

**Step 3 .**

The weight of each DCT block is determined through the Euclidean distance of the Gaussian model. And the *r*^*th*^ feature of the feature map is processed through the following equation [14]:

(4) $$\begin{array}{c} G_{m}^{r}=\sum_{m\neq n}\frac{1}{\sigma \sqrt{2\pi }}e^{-\frac{d_{m,n}^{2}}{2\sigma^{2}}D_{m,n}^{r}}. \end{array}$$

In the above equation,  *G*_*m*_^*r*^ stands for the obtained significance value through r_th_;  *σ* refers to the Gaussian model parameters, and  *σ*=5; *d*_*m*,*n*_ accords to the European distance between *m*, *n* in the DCT block.

**Step 4 .**

The feature map is fused by the coherent normalization method to obtain the significance map [15, 16]. The calculation method of significance diagram is shown as follows:

(5) $$\begin{array}{c} G=\sum^{}\varphi_{\vartheta }L\left(\vartheta \right)+\omega \prod L\left(\vartheta \right). \end{array}$$

In the above equation, *L* represents the normalization operation;  *ϑ*,  *φ*_*ϑ*_, *ω* denotes the weight of each component, and *φ*_*ϑ*_=*ω*=1/5. The significance diagram can be obtained through the above steps.  Figure 2 depicts the specific non peer-to-peer encryption process.

#### 3.1.2. Important Area Encryption

Here, dynamic DNA combined with the chaotic encryption algorithm is used to encrypt important areas in video images, which has strong confidentiality [17–19]. There are four nucleic acids A, T, G, and C in the DNA sequence, and their coding rules are shown in Figure 3.

The image encryption process can be realized by disrupting the DNA encoding and decoding of each pixel, and the data encryption performance can be improved by introducing some algebraic operations for DNA sequences [20, 21]. Figures 4, 5, and 6 describe the XOR and addition and subtraction operations of DNA series.

The key used in this scheme is a pseudorandom sequence generated by a four-dimensional chaotic system. Equation (6) manifests the calculation equation of the system:

(6) $$\begin{array}{c} \left\{\begin{array}{c} \dot{x}=a\left(y-x\right)+w,\\ \dot{y}=cx-y-2xz,\\ \dot{z}=2x^{2}-bz,\\ \dot{w}=yz-dw. \end{array}\right. \end{array}$$

In the above equation, *x*, *y*, *z*, *w* represent the state variables; *a*, *b*, *c*, *d* denote the system parameters; when *a*=10, *b*=8/3, *c*=28, *d*=2, the four-dimensional chaotic system is in the hyperchaotic state [22]. The encryption steps of important areas are as follows:

**Step 5 .**

A random matrix is generated through iterative logical mapping, which is the same size as the important area in the video image. Equation (7) illustrates the calculation method of iterative logical mapping:

(7) $$\begin{array}{c} \mu_{n+1}=\lambda \mu_{n}\left(1-\mu_{n}\right). \end{array}$$

In the above equation, *λ* stands for *p* parameters; *μ*_0_ means the calculation method of the first term of the recurrence, which is shown in the equation as follows:

(8) $$\begin{array}{c} \mu_{0}=\frac{1}{I\times J\times 255}\sum_{m=1,n=1}^{I,J}P\left(m,n\right). \end{array}$$

In the above equation, *I* × *J* represents the size of the original video image; *P* indicates the original video image; (*m*, *n*) denotes the pixel position in the original video image; *P*(*m*, *n*) expresses the pixel value.

**Step 6 .**

For the important area *Gx* and random matrix *φ*(*x*), their pixel values of DNA sequence are converted to binary, and the important region and random matrix are encoded according to the coding rules of DNA sequence [23].

**Step 7 .**

Four key sequences *x*_*n*_, *y*_*n*_, *z*_*n*_, *w*_*n*_ are generated by the chaotic system. Since it contains the coding rules of DNA sequences in (8), it is necessary to pair the keys *x*_*n*_, *y*_*n*_ through the following equation:

(9) $$\begin{array}{c} \left\{\begin{array}{c} x_{n}=mod\left(\left[x_{n}\times 10^{5}\right],8\right),\\ \left.y_{n}=mod\left(|y_{n}\times 10^{5}\right],8\right). \end{array}\right. \end{array}$$

In the above equation, there are 8 possibilities for the value of *x*_*n*_, *y*_*n*_. The keys *x*_*n*_, *y*_*n*_ convert important regions and random matrix sequences into DNA sequences.

**Step 8 .**

The DNA sequence includes three operations: XOR, addition, and subtraction. The key *z*_*n*_ is processed by the DNA operation [24]. Equation (10) demonstrates the calculation method:

(10) $$\begin{array}{c} z_{n}=mod\left(\left[z_{n}\times 10^{5}\right],3\right). \end{array}$$

In the above equation, there are three possibilities for the value of the key *z*_*n*_, and the operation rules of the DNA sequence can be obtained by the key *z*_*n*_. Through DNA manipulation, the DNA sequences of important regions and random matrices are processed to obtain encrypted DNA sequences.

**Step 9 .**

The key *w*_*n*_ is processed through the equation as follows:

(11) $$\begin{array}{c} w_{n}=mod\left(\left[w_{n}\times 10^{5}\right],8\right). \end{array}$$

When the form of the DNA sequence is transformed from binary to decimal, the encrypted image of the important area can be obtained. The encryption process and decryption process are inverse to each other.

#### 3.1.3. Nonimportant Area Encryption

Here, the compressed sensing (CS) algorithm is used to encrypt the nonimportant area of the video image. A compressed sensing algorithm can encrypt and protect the video image and compress the video image.

In certain cases, the original signal can be accurately restored by partial sampling data. If a one-dimensional discrete-time signal *w*of length*Q* is compressed and projected, a measurement matrix *P* × *Q*(*P* “*Q*) can be combined with Bernoulli Gaussian random matrix or partial Adama matrix. Equation (12) demonstrates the process as follows:

(12) $$\begin{array}{c} v=\theta \omega . \end{array}$$

In the above equation, *v* represents the one-dimensional compressed measurement vector, whose size is *P* × 1. When the signal *ω* is not sparse, it can be represented by the equation as follows:

(13) $$\begin{array}{c} \omega =\xi x. \end{array}$$

In the above equation, *ξ* denotes the sparse orthogonal basis, whose size is *Q* × *Q*; *x* indicates the parse vector.

Equation (14) illustrates the sampling process of compressed sensing:

(14) $$\begin{array}{c} v=\theta \xi x=\Psi x. \end{array}$$

In the above equation, Ψ=*ξx* stands for the sensing matrix of compressed sensing, whose size is *P* × *Q*(*P* “*Q*).

In the compression sensing sampling process, it is relatively easy to get the measured value *v* from the original value *ω*, while the probability is very small to get the original signal *ω* from the measured value *v* because the inverse sampling process of compressed sensing has countless solutions.

When the measured value *v* and matrix Ψ meet certain conditions, and the sparsity of the vector *x* is strong, the measured value *v* is transformed to the optimization problem of the original signal *ω*. Equation (15) illustrates the process as follows:

(15) $$\begin{array}{c} Minimize||x{||}_{0}subject\;to\;v=\Psi x. \end{array}$$

In the above equation, ||*x*||_0_— *x* stands for the norm of *L*_0_.

By solving the optimization problem, the original value can be rebuilt as $\hat{\omega }=\xi \hat{x}$. A semitensor product (STP) is introduced in the compressed sensing process. Its definition is shown as follows:

(16) $$\begin{array}{c} S=M\times N. \end{array}$$

In the above equation,  *M* *and* *N* mean matrixes, and *M* ∈ *R*^*a*×*b*^, *N* ∈ *R*^*c*×*d*^; *S* stands for the semitensor convolution of *M* *and* *N*.

The factor of *c*(*c*=*bt*) is set as *b*, and *m*_*ab*_ ∈ *M*, *n*_*cd*_ ∈ *N* so that the following equation can be obtained as

(17) $$\begin{array}{c} T=\left[\begin{array}{ccc} m_{11} & \ldots & m_{1b}\\ \vdots & \ddots & \vdots \\ m_{a1} & \ldots & m_{ab} \end{array}\right]\times \left[\begin{array}{ccc} n_{11} & \ldots & n_{1d}\\ \vdots & \ddots & \vdots \\ n_{c1} & \ldots & n_{cd} \end{array}\right]=\left[\begin{array}{ccc} m_{11} & \ldots & m_{1b}\\ \vdots & \ddots & \vdots \\ m_{a1} & \ldots & m_{ab} \end{array}\right]\times \left[\begin{array}{ccc} N^{11} & \ldots & N^{1d}\\ \vdots & \ddots & \vdots \\ N^{b1} & \ldots & N^{bd} \end{array}\right]. \end{array}$$

In the above equation, *n*_*ab*_(*a*=1,2, ⋯, *c*; *b*=1,2, ⋯, *d*) refers to the result obtained after the division is conducted on the *jth* column in matrix *N*. *N*^*ab*^ indicates the column vector with a length of *t*. When *b*=*c* and *M* × *N*=*MN*, the STP is reduced to the traditional matrix product.

*P* × *Q* and *Q* × *Q* are the sizes of measurement matrix and original video image matrix in traditional compressed sensing, *P* × *Q* is the size of the encrypted video image in compressed sensing, and *P*/*Q* represents the compression ratio of compressed sensing. The smaller the value of *P*/*Q*, the smaller the storage of video images. When large data images need to be processed, certain storage resources can be saved. While if the value of *P*/*Q* is too small, the original video image will be distorted. Therefore, it is necessary to find the balance between video image restoration and compression ratio. There are three main steps to compress unimportant areas in the video image, as shown in Figure 7.

### 3.2. Neural Network

Two obvious properties of the backpropagation (BP) algorithm determine its computing power: first, the local calculation of the algorithm is relatively simple; second, when online learning is carried out step by step, the descent of the random gradient can be realized in the parameter space. The BP algorithm provides theoretical support for the development of supervised training and learning [25]. When neuron *j* is output, the induced local domain through the activation function is shown as follows:

(18) $$\begin{array}{c} v_{j}\left(n\right)=\sum_{i=0}^{m}w_{j}\left(n\right)y_{i}\left(n\right). \end{array}$$

In the above equation, *y*_*i*_(*n*) means the calculated value in the neuron *j*, which is determined by the excitation generated by the upper layer. Therefore, the error value obtained from the neuron *j* can be recorded as follows:

(19) $$\begin{array}{c} e_{j}\left(n\right)=d_{j}\left(n\right)-y_{j}\left(n\right). \end{array}$$

In the above equation, *d*_*j*_(*n*) stands for *d*(*n*) elements in neuron *j*.

The resulting instantaneous error energy can be expressed as *ξ*_*j*_(*n*)=1/2*e*^2^(*n*). By accumulating the excitation error energy generated by the whole neuron, the instantaneous error energy generated by the whole neural network can be obtained as follows:

(20) $$\begin{array}{c} \xi \left(n\right)=\underset{j\in C}{\sum }\xi_{j}\left(n\right)=\frac{1}{2}\underset{j\in C}{\sum }e^{2}\left(n\right). \end{array}$$

In the above equation, *C* denotes the set that contains all neurons in the output layer. If the dataset contains *N* examples, then the following equation illustrates the empirical risk of the dataset:

(21) $$\begin{array}{c} \xi_{\alpha v}\left(N\right)=\frac{1}{N}\sum_{n=1}^{N}\xi \left(n\right)=\frac{1}{2N}\overset{N}{\underset{n=1}{\sum }}\underset{j\in C}{\sum }e_{j}^{2}\left(n\right). \end{array}$$

So, when the iterated quantity is *n*, equation (22) expresses the calculation of the final output value of neuron *j* excitation occurred on *y*_*j*_(*n*):

(22) $$\begin{array}{c} y_{j}\left(n\right)=\varphi_{j}\left(v_{j}\left(n\right)\right). \end{array}$$

BP algorithm differentiation uses $w_{j\dot{n}}\left(n\right)$ on the parameters, which is related to partial derivative ∂*ξ*(*n*)/∂*w*_*jμ*_(*n*). In the direct proportion, using chain iteration, the gradient can be written as follows:

(23) $$\begin{array}{c} \frac{\partial \xi \left(n\right)}{\partial w_{ji}\left(n\right)}=\frac{\partial \xi \left(n\right)}{\partial e_{j}\left(n\right)}\frac{\partial e_{j}\left(n\right)}{\partial y_{j}\left(n\right)}\frac{\partial y_{j}\left(n\right)}{\partial v_{j}\left(n\right)}\frac{\partial v_{j}\left(n\right)}{\partial w_{j_{j}}\left(n\right)}. \end{array}$$

In the above equation, ∂*ξ*(*n*)/∂*w*_*ji*_(*n*) refers to the update degree of *p* parameters in the parameter data *w*_*ji*_.

*e*_*j*_(*n*) in (20) is used to obtain the following equation:

(24) $$\begin{array}{c} \frac{\partial \xi \left(n\right)}{\partial e_{j}\left(n\right)}=e_{j}\left(n\right). \end{array}$$

*y*_*j*_(*n*) in (19) is used to obtain the following equation:

(25) $$\begin{array}{c} \frac{\partial e_{j}\left(n\right)}{\partial y_{j}\left(n\right)}=-1. \end{array}$$

*v*_*j*_(*n*) in (22) is used to obtain the following equation:

(26) $$\begin{array}{c} \frac{\partial y_{j}\left(n\right)}{\partial v_{j}\left(n\right)}=\varphi_{j}^{\text{'}}\left(v_{j}\left(n\right)\right). \end{array}$$

*w*_*ji*_(*n*) in (18) is used to obtain the following equation:

(27) $$\begin{array}{c} \frac{\partial v_{j}\left(n\right)}{\partial w_{ji}\left(n\right)}=y_{i}\left(n\right). \end{array}$$

Equations (24)–(27) are replaced into (23) to obtain the following equation:

(28) $$\begin{array}{c} \frac{\partial \xi \left(n\right)}{\partial w_{ji}\left(n\right)}=-e_{j}\left(n\right)\varphi_{j}^{\text{'}}\left(v_{j}\left(n\right)\right)y_{i}\left(n\right). \end{array}$$

Equation (29) manifests the process of the correction of *w*_*ji*_(*n*) for the $w_{j\dot{n}}\left(n\right)$ corresponding to the delta rule:

(29) $$\begin{array}{c} \Delta w_{ji}\left(n\right)=-\eta \frac{\partial \xi \left(n\right)}{\partial w_{ji}\left(n\right)}. \end{array}$$

In the above equation, *η* refers to the learning rate parameter of the BP algorithm; “−” indicates the gradient descent during the search for parameters.

Equation (28) is transformed into (29) to obtain the following equation:

(30) $$\begin{array}{c} \Delta w_{ji}\left(n\right)=\eta \delta_{j}\left(n\right)y_{i}\left(n\right). \end{array}$$

The local gradient *δ*_*j*_(*n*) is defined as

(31) $$\begin{array}{c} \delta_{j}\left(n\right)=\frac{\partial \xi \left(n\right)}{\partial v_{j}\left(n\right)}=\frac{\partial \xi \left(n\right)}{\partial e_{j}\left(n\right)}\frac{\partial e_{j}\left(n\right)}{\partial y_{j}\left(n\right)}\frac{\partial y_{j}\left(n\right)}{\partial v_{j}\left(n\right)}=e_{j}\left(n\right)\varphi_{j}^{\text{'}}\left(v_{j}\left(n\right)\right). \end{array}$$

The above equation reveals that for the excitation local gradient *δ*_*j*_(*n*) of the neurons *j* and its error value *e*_*j*_(*n*) and activation function derivative *φ*_*j*_′(*v*_*j*_(*n*)), their product of values is consistent. Combined with (30), it can be seen that the error value of excitation *e*_*j*_(*n*) of the neurons *j* plays a decisive role in the date parameters $w_{j\dot{n}}\left(n\right)$ [26, 27].

### 3.3. Password Security Detection Method

In this section, a numerical conversion operator is added to the adversarial encryption network structure to enable the adversarial neural network to learn a specific form of the cryptographic algorithm and form a relatively simple structure to reason the security of the encrypted block cipher. Exclusive OR (XOR) is a well-known binary nondifferentiable operation often used in cryptography. This paper uses a continuous generalization of the operator XOR.

It is essential to generalize the XOR operation to realize a neural network that can perform an internal XOR. The XOR operation can be generalized with the unit circle by mapping bit 0 to corner 0 and bit 1 to corner *π* so that XOR is equal to the sum of the two corners.

However, since the sum is a continuous operation, angles other than 0 or *π* can be used in the calculation process. To generalize it to a continuous space, the mapping of bit *b* to angle is defined as

(32) $$\begin{array}{c} f\left(b\right)=\text{arccos}\left(1-2b\right). \end{array}$$

The inverse operation of *f* provides the mapping between the angle *a* to a consecutive bit as

(33) $$\begin{array}{c} f^{-1}\left(a\right)=\frac{1-\text{cos}\left(a\right)}{2}. \end{array}$$

With this operator, this paper can learn to verify the security degree of encryption by introducing a small neural network called an encryption detection network, as presented in Figure 8.

The encryption detection network receives plaintext and key as input. For each received plaintext and key, the transformation defined in (32) is applied to convert the bit information into angle information as the neural network input. Then, a weight matrix multiplication of the adversarial encryption network is employed to obtain the corresponding preliminary ciphertext. Besides, the final ciphertext is obtained through the inverse transformation defined in (33). It should be noted that the encrypted detection network is the same as other neural networks, and the data processed are all floating-point numbers. Consequently, the ciphertext of the encrypted detection network is not composed of bits but composed of floating-point numbers between 0 and 1.

Mathematically speaking, the fully connected layer of the cipher set performs the following operations:

(34) $$\begin{array}{c} {\left(\begin{array}{c} h_{0}\\ h_{1}\\ \vdots \\ h_{n-1} \end{array}\right)}^{T}={\left(\begin{array}{c} a_{0}\\ \vdots \\ a_{n-1}\\ a_{n}\\ \vdots \\ a_{2n-1} \end{array}\right)}^{T}W. \end{array}$$

In the above equation, *W* denotes the unified definition of the weight matrix of all hidden layers and convolutional layers in the adversarial encryption network, *a*_0_,…, *a*_2*n*−1_ represents the angle obtained from the plaintext and the key, and *h*_0_, ..., *h*_*n*−1_ refers to the output variable of the antiencryption network.

In the following sections, this paper mathematically represents the cipher set as a function:

(35) $$\begin{array}{c} C=\xi_{n}\left(W,P,K\right). \end{array}$$

In the above equation, *W* stands for the weight matrix, and *P*, *K*, and *C* are the *n*-bit vector of the input plaintext, the key, and the output ciphertext, respectively.

Cipher sets can learn to combine inputs in several ways. Since the input bits are mapped to corner 0 or *π*, if all the concatenated values ( *W* elements) are integers, then the result will be equivalent to an XOR operation of the input bits. Due to the random initialization of all weights, the probability that the weight elements are integers is close to 0. Therefore, this paper can use this model to analyze the security of encrypted data and make inferences.

### 3.4. Improved Antineural Network Encryption Algorithm Based on CCA

#### 3.4.1. Loss Function Design

Primarily, Bob and Alice encrypt and decrypt against the encrypted network. The attacker Eve's network structure needs to be improved. The adjusted Eve is a classifier and will receive C, K1, and K0. If the attacker thinks K_If 0 is the source of C, C will be classified as 0, but if the attacker thinks that K_If 1 is the source of C, C will be classified as 1.  Figure 9 manifests the network settings of Eve.

The eve neural network designed here will receive and convert the bits *C*,  *K*_1_, *K*_0_ into angles by

(36) $$\begin{array}{c} f\left(b\right)=arccos\left(1-2b\right). \end{array}$$

The generalized XOR operation constitutes each rule, which is converted into continuous bits by

(37) $$\begin{array}{c} f^{-1}\left(a\right)=\frac{1-cos\left(a\right)}{2}. \end{array}$$

The results obtained are merged into the logic passing through the softmax layer through the second fully connected layer; thus the ciphertext of*K*_0_is obtained as probability *k*_0_(*C*). The ciphertext of *K*_1_ is probability *k*_1_(*C*). If *k*_1_ > *k*_0_, the output is 0; otherwise, the output is 1.

In Figure 9, the attacker Eve will receive *K*_1_,  *K*_0_ two keys and ciphertext *C* and sends the key *K*_1_, *K*_0_ as input. [*k*_1,0_,…, *k*_1,*n*−1_] represents the key *K*_1_, [*k*_0,0_,…, *k*_0,*n*−1_] rrepresents the key *K*_0_. [*c*_0_,…, *c*_*n*−1_] indicates the ciphertext *C*. The orientation angle can be adjusted by equation (36). For conversion, the adoption of angle information can generate a full connection layer [*h*_0_^1^, *h*_1_^1^,…, *h*_*R*−1_^1^] of this hidden variable, where *R* represents the number of neurons in the hidden layer. Equation (37) converts the angle information into $\left[h_{0}^{1},h_{1}^{1},\ldots ,h_{\bar{R}-1}^{1}\right]$. For this continuous bit information, the values of all continuous bit information are in the interval [0, 1] [28–30]. The variables in the hidden layer can be introduced into the classification logic through another fully connected layer, and the final output result is as follows: Ciphertext *C* generated by key *K*_1_ and probability *π*_1_, and ciphertext *C* generated by key *K*_0_ and probability *π*_0_.

Due to the change of the model, the loss function of Eve needs to be redefined to optimize the problem to adapt to the new countermeasure network model. To do this, the preset keys are [*k*_0_^(0)^, *k*_0_^(1)^,…, *k*_0_^(*M* − 1)^], [*k*_1_^(0)^, *k*_1_^(1)^,…, *k*_1_^(*M* − 1)^], and a ciphertext [*C*^(0)^, *C*^(1)^,…, *C*(*M* − 1)]. Equation (38) signifies the definition of the loss of Eve:

(38) $$\begin{array}{c} L_{E}=-\frac{1}{M}\overset{M-1}{\underset{i=0}{\sum }}\overset{1}{\underset{j=0}{\sum }}t_{j}^{\left(i\right)}\text{log}\left(\pi_{j}^{\left(j\right)}\right). \end{array}$$

In the above equation, *C*^(*i*)^ denotes the ciphertext generated by key *P*_0_^(*i*)^, *t*_1_^(*i*)^=1, or *t*_1_^(*i*)^=0. Therefore, the attacker Eve learns by minimizing *L*_*E*_, while Bob and Alice learn by minimizing the given  *L*. Equation (39) demonstrates the specific process as follows:

(39) $$\begin{array}{c} L=L_{AB}-\gamma min\left(Err,0.5\right). \end{array}$$

In the above equation, *Err* indicates the classification error of Eve; *γ* represents the super parameter.

#### 3.4.2. Model Structure Design

In the new countermeasure network model, Eve will choose *K*_1_, *K*_0_ two keys and sends them to Alice. Alice will choose one of the two keys and encrypt it through a neural network to get the ciphertext *C* and put the obtained ciphertext *C* to Bob and Eve. Bob will use the key and ciphertext to decrypt the information through the neural network, but Eve will not decrypt the cracked ciphertext *C* to attack but will judge the encryption of the key through the neural network, and then output 0 or 1 according to the judgment result. This model is called the CCA-ANC model. In the CCA-ANC model, Bob and Alice need to communicate through a better encryption system to ensure the security of the communication process.  Figure 10 illustrates the specific model structure.

#### 3.4.3. Experimental Simulation Parameter Setting

This paper uses a Mini-batch of which *M*= 4096 and *γ*=7 to train the network. The L2 regularization method is also used in the experiment, where the key length is 4 bits (*n*=4); the 8 bit (*n*=8) hyperparameter *α*=0.1; the key length is 16 bits ( *n*=16); the hyperparameter *α*=0.015. Meanwhile, for the Eve network, this paper defines the number of neurons in the hidden layer as *R*=4*n*. Then, Eve can simultaneously analyze the number of linear combinations of functions. With the increase of the key size, Eve needs more function calculation formulas. Therefore, this paper chooses these parameters according to experience and sets them in proportion to the number of bits of the key, increasing the number of linear combinations. In this way, Eve can crack the password learned by Alice and Bob through the neural network.  Table 1 reveals the relevant learning parameters of the algorithm model.

## 4. Simulation Experiment and Data Analysis

### 4.1. Security Analysis of Attacker-Free Algorithm

In the present work, equation (36) is used to test the nonattack model.  Figure 11 presents the results.

Figure 10 manifests that the communication between Bob and Alice is error free, so all experiments are successful, but the encryption algorithm used in all experiments does not have strong security. For example, equation (40) expresses the encryption algorithm in an experiment:

(40) $$\begin{array}{c} \xi_{n}\left(W_{ronud\;},P,K\right)={\left[\begin{array}{c} p_{1}\\ p_{0}\\ p_{6}\\ p_{3}\\ p_{4}\\ p_{5}\\ p_{2}\\ p_{7} \end{array}\right]}^{T}. \end{array}$$

In the above equation, there is *P*=[*p*_0_, *p*_1_,…, *p*_7_], *K*=[*k*_0_, *k*_1_,…, *k*_7_]. The learning algorithm of (40) does not use the encryption key, and these experiments do not produce a secure encryption system. The reason for this phenomenon is that Bob and Alice are trained without any security problems. In the process of communication through the encrypted network, they do not require the encryption effect but only ensure its accuracy.

### 4.2. Security Analysis of ANC Algorithm

The minimization function is used to ensure that Alice and Bob do not try to maximize Eve's error so that Eve can flip all the bits in the next round and get a correct guess. If Eve guesses the plaintext, it would expect about half the correct bits, with an average error of 0.5, as shown in Figure 12.

During the experiment, in addition to using 16 bit plaintext and ciphertext for training, this paper also uses 8 bit and 4 bit plaintexts and keys for training, and the results are shown in Figure 13.

Figure 13 demonstrates that the model's training speed and antiencryption effect continue to increase with the growth of the plaintext and the key. The reason is that when the key and the plaintext grow, the hidden units in the neural network can train more complex functions to meet the loss function's requirements. Therefore, the neural network encryption model is suitable for encrypting long block plaintext. However, since it is impossible to detect whether the encrypted ciphertext uses a key to encrypt the plaintext, the ANC encryption algorithm still has security flaws.

The present work tests the learned encryption network through (36), as shown in Figure 14.

After the training of Bob and Alice, because a relatively simple antiencryption structure is obtained from the training, its security can be simply described without the help of a neural network. So, the present work does not continue to train Eve. Figure 14 indicates the training results. If the communication between Bob and Alice during the execution of (36) in each experiment is correct, the learning model can be considered to be successful. If an antiencryption network can be encrypted by different functional methods, it can be considered to be secure. For example, equation (41) illustrates the password learned by Bob and Alice.

(41) $$\begin{array}{c} \xi_{n}\left(W_{rownd\;},P,K\right)={\left[\begin{array}{c} p_{0}⊕k_{3}\\ p_{3}⊕k_{0}\\ p_{2}⊕k_{0}⊕k_{3}⊕k_{4}⊕k_{5}⊕k_{6}⊕k_{7}\\ p_{1}⊕k_{0}\\ p_{4}⊕k_{1}\\ p_{5}⊕k_{2}\\ p_{6}⊕k_{2}\\ p_{7}⊕k_{1} \end{array}\right]}^{T}. \end{array}$$

In this antiencryption network, the communication between Bob and Alice is error free, so it can be considered that it is a success of the design training of the network. However, the security of this encryption method is poor because several plaintext bits are encrypted with the same key bit. According to the training results, since the generation of plaintext is irregular, all attackers with Eve knowledge cannot recover the plaintext. If there is *c*_1_ = *c*_3_ = 0, then there is supposed to be *c*_1_ ⊕ *c*_3_ = *p*_1_ ⊕ *p*_3_, and *p*_1_ = *p*_3_ exists when bits are encrypted with the same key bit. Using Eve to predict the best *p*_1_, *p*_3_ result is that the two parameters have the same value. Eve can predict two bits rightly or wrongly in half the time by adopting this strategy.

### 4.3. Security and Efficiency Analysis of CCA-ANC Algorithm

If Bob and Alice can ensure the accuracy of the communication process during the implementation of the algorithm in the experiment, the learning and training model can be considered as successful; otherwise, the learning and training model is considered as a failure. If Eve cannot extract information from the ciphertext, it can be considered that a trained encryption countermeasure network is secure for Eve. For example, in a confrontation network learning, Bob and Alice get two cryptosystems. When *n* = 8, the arbitrarily selected training result analysis is obtained as shown as follows:

(42) $$\begin{array}{c} \xi_{u}\left(W_{ronud\;},P,K\right)={\left[\begin{array}{c} p_{0}⊕k_{7}\\ p_{1}⊕k_{5}\\ p_{2}⊕k_{6}\\ p_{3}⊕k_{0}\\ p_{4}⊕k_{1}\\ p_{5}⊕k_{4}\\ p_{6}⊕k_{3}\\ p_{7}⊕k_{2} \end{array}\right]}^{T}. \end{array}$$

When *n*=16, equation (43) manifests the analysis of arbitrarily selected training results:

(43) $$\begin{array}{c} \xi_{n}\left(W_{round\;},P,K\right)=\left[\begin{array}{c} p_{0}\;⊕\;k_{8}\\ p_{1}\;⊕\;k_{7}\\ p_{2}\;⊕\;k_{0}\\ p_{3}\;⊕\;k_{3}\\ p_{4}\;⊕\;k_{11}\\ p_{5}\;⊕\;k_{9}\\ p_{6}\;⊕\;k_{2}\\ p_{7}\;⊕\;k_{6}\\ p_{8}\;⊕\;k_{15}\\ p_{9}\;⊕\;k_{13}\\ p_{10}\;⊕\;k_{1}\\ p_{11}\;⊕\;k_{5}\\ p_{12}\;⊕\;k_{4}\\ p_{13}\;⊕\;k_{14}\\ p_{14}\;⊕\;k_{12}\\ p_{15}\;⊕\;k_{10} \end{array}\right]. \end{array}$$

Equations (42) and (43) manifest that Bob and Alice's encrypted network trained and learned has certain security.  Figure 15 manifests the average test results.

In the experimental testing process of the present work, there are only two failures in the training and learning results of models. The communication between Bob and Alice could not be carried out smoothly. Most of the training models have successfully trained and learned the secure encryption network under the proposed CCA-ANC method, and only a few training models have not learned the secure encryption network due to the randomness of neural network and key length. After comparing Figures 14 and 15, it can be found that there is an increase in the number of successful experiments. Through the experimental results, it can be found that Eve has a strong decoding ability in the original encryption method of ANC, and it obtains relatively less information. It is difficult to crack only the pure secret translation. Therefore, Bob and Alice have more encryption solutions to choose from, the selection space is also large, and the objective function trained by ANC will be more complex. The CCA-ANC encryption method is trained and cracked through the neural network. To ensure the security of communication results, the only way Bob and Alice can take is to find a more secure solution that cannot be cracked by attacker Eve. Therefore, compared with the original ANC model, the objective function has a better effect.  Figure 16 illustrates the training results of the CCA-ANC.

Eve's intention is to maximize the classification accuracy, while Bob and Alice's intention is to minimize Bob's decryption error value and Eve's classification accuracy.  Figure 16 illustrates that when Bob's decryption error rate decreases, the average classification error rate of Eve will increase over time; while when Bob and Alice learn a secure encryption network structure, Eve's classification accuracy is not superior to random prediction. The encryption effect of the ANC algorithm is still better when the key length is shortened.

To test the encryption efficiency of the CCA-ANC encryption algorithm, 1024 MB data is input to test for encryption speed of data encryption standard (DES), 3DES, advanced encryption standard (AES), and CCA-ANC simultaneously.  Figure 17 depicts the test results.

After the neural network training, the neural network model will receive data input, most of which are linear data operations, with fast speed.  Figure 17 demonstrates that the encryption time of CCA-ANC is 14s and the average speed is 69 Mb/s, which has obvious advantages over other encryption algorithms.

## 5. Conclusions

With IoT, big data, and social networks rising, the storage and sharing of digital video images have been deeply involved in all aspects of people's life. The food images stored and shared by the cloud platform often contain a large amount of private information of users. The leakage of this information has a significantly negative impact on the personal life and seriously hinders the healthy development of social media and cloud platform services. To prevent the disclosure of users' privacy and ensure the safe storage and sharing of video image data in the cloud platform, what is proposed is an encryption algorithm against neural cryptography. Initially, the image saliency detection algorithm is used to identify the significant target of the video image. According to the significant target, the important region and nonimportant region are divided adaptively, and the encrypted two regions are reorganized to obtain the final encrypted image. Then, by introducing the attacker who uses the ciphertext mode to conduct criminals, what is proposed is an improved encryption algorithm based on selective ciphertext attack. Besides, to improve the existing encryption algorithm of the neural network, a secure encryption algorithm is obtained through detailed analysis and comparison of the security ability of the algorithm. By comparing the encryption efficiency of different encryption algorithms, it is concluded that the CCA-ANC algorithm constructed here takes 14s for encryption, and the average speed is 69 MB/s. Therefore, this model has obvious advantages compared with other encryption algorithms.

Using the CCA-ANC algorithm proposed here, all models learned in the long key can be guaranteed to be secure. But when attackers use more powerful technologies to forcibly integrate the solution into a powerful encryption system, only using the CCA-ANC method is not enough to ensure the security of information. Designing an adversary attacker with a strong ability to prevent attacks on the cryptosystem is the key to guaranteeing the performance of the algorithm. In future work, more experiments will be carried out to evaluate more parameters. Simultaneously, it is necessary to implement a parallel way to improve the performance of the algorithm and use larger keys and attackers with stronger attack ability to improve the model.

## Figures and Tables

**Figure 1:** Algorithm steps.

**Figure 2:** Non peer encryption flow.

**Figure 3:** DNA coding rules.

**Figure 4:** XOR operation of DNA sequences.

**Figure 5:** Addition of DNA sequences.

**Figure 6:** Subtraction of DNA sequences.

**Figure 7:** Compression process of unimportant areas.

**Figure 8:** Encryption detection network.

**Figure 9:** Eve neural network.

**Figure 10:** CCA-ANC model.

**Figure 11:** Key learning and test results of different sizes.

**Figure 12:** Training results of ANC by the 16 bit plaintext.

**Figure 13:** Training results of ANC by 4 bit and 8 bit plaintexts: (a) 4 bit plaintext; (b) 8 bit plaintext.

**Figure 14:** ANC algorithm learning and testing neural network.

**Figure 15:** Test results of 50 neural networks using CCA-ANC.

**Figure 16:** Training results of CCA-ANC (a: 4 bit; b: 8 bit; c: 16 bit).

**Figure 17:** Comparison of encryption efficiency of different encryption algorithms.

**Table 1:** Parameters of the CCA-ANC algorithm.

Model settings	Parameter
Mini-batch	4096
Optimizer	Adam
Learning rate	0.0008
Key length	16, 8, 4

## Data Availability

The data used to support the findings of this study are included within the article.
